RETRACTED

# Perceptual load affects spatial tuning of neuronal populations in human early visual cortex

**DOI:** 10.1016/j.cub.2013.11.061

**Published:** 2014-01-20

**Authors:** Benjamin de Haas, D. Samuel Schwarzkopf, Elaine J. Anderson, Geraint Rees

**Affiliations:** 1 Institute of Cognitive Neuroscience, University College London, Alexandra House, 17 Queen Square, London WC1N 3AR, UK; 2 Wellcome Trust Centre for Neuroimaging, University College London, Alexandra House, 17 Queen Square, London WC1N 3AR, UK; 3 Cognitive Perceptual and Brain Sciences, University College London, Alexandra House, 17 Queen Square, London WC1N 3AR, UK; 4 Institute of Ophthalmology, University College London, Alexandra House, 17 Queen Square, London WC1N 3AR, UK

## Abstract

Withdrawal of attention from a visual scene as a result of perceptual load modulates overall levels of activity in human visual cortex [1], but its effects on cortical spatial tuning properties are unknown. Here we show attentional load at fixation affects the spatial tuning of population receptive fields (pRFs) in early visual cortex (V1–3) using functional magnetic resonance imaging (fMRI). We found that, compared to low perceptual load, high perceptual load yielded a ‘blurrier’ representation of the visual field surrounding the attended location and a centrifugal ‘repulsion’ of pRFs. Additional data and control analyses confirmed that these effects were neither due to changes in overall activity levels nor to eye movements. These findings suggest neural ‘tunnel vision’ as a form of distractor suppression under high perceptual load.

## Main Text

Load theory [2] proposes that increasing processing load associated with an attended target will suppress perceptual processing of distractors due to progressive exhaustion of fixed processing capacity. Consistent with this, high target-associated perceptual load reduces distractor-related interference in response competition tasks [3], it diminishes visual sensitivity [4] and adaptation [5] to distractors, and reduces overall responses to distractors in human visual cortex [1]. However, it is unclear whether perceptual load affects other fundamental properties of neuronal processing, such as the spatial preference of neuronal populations in human early visual cortex.

We used pRF mapping [6] to estimate spatial tuning functions of neuronal populations throughout human V1–3 under high *versus* low perceptual load conditions. The pRF is defined as the location and spatial extent of positions in the visual field where stimulation evokes responses that can be measured using fMRI at a corresponding visual cortex location (voxel).

Participants performed a task of either high or low perceptual load on identical streams of stimuli presented at central fixation while task-irrelevant mapping stimuli traversed the visual field (Figure 1A). The task-irrelevant stimuli were used to infer the size and location of pRFs. We found that high (versus low) perceptual load in the central task significantly affected the spatial tuning of early visual cortex for the surrounding visual field (Figure 1B–D). For every voxel with pRF centre position from 1–7 degrees eccentricity we calculated the relative size difference of its pRF under high *versus* low load.

RETRACTED

**Figure 1:** Effect of perceptual load on spatial tuning of neuronal populations. (A) The fixation task required detection of targets in a rapid series of coloured upright or inverted crosses (c.f. Schwartz *et al*. [1]). Targets were defined on colour alone (low load) or the conjunction of colour and orientation (high load). Target frequency and stimulus streams were identical between conditions. Task-irrelevant bar-type mapping stimuli traversed the surrounding visual field. Participants were significantly less sensitive (t_25_ = 11.83, *P* < 10^–11^) and slower (t_25_ = 15.75, *P* < 10^–13^) when detecting high versus low load targets, indicating successful manipulation of perceptual load. (B) pRF size by eccentricity, visual area and condition. pRF sizes increased with eccentricity and along the visual hierarchy. From 3.5 to 6.5 degrees eccentricity perceptual load affected pRF size estimates, with bigger pRFs under high (red) vs. low (black) perceptual load. Lines and error shades indicate sample mean ± one standard error of the mean (s.e.m.). Line styles indicate visual area (see inset). (C) Effect of high *versus* low perceptual load on pRF size. Relative size differences between conditions were computed and expressed as % size difference. Positive values indicate bigger pRFs under high vs. low perceptual load. Error shades indicate ± one s.e.m. Colour indicates visual area (see inset). (D) Effect of high *versus* low perceptual load on pRF eccentricity. Eccentricity differences between conditions were computed and normalised by pRF size (under low load; expressed as % of pRF size). Positive values indicate an outward pull of pRFs under high vs. low perceptual load. Error shades indicate ± one s.e.m. Colour indicates visual area (see inset). Data for all plots were binned according to pRF centre eccentricities as determined in the low load condition (thus comparing pRFs of identical voxels; see Supplemental Methods for details).

We found that pRF size significantly increased under high perceptual load across participants and hemispheres for V1 (mean increase = 12.31% ± s.e.m. = 4.14%, *t*_48_ = 2.97, *PFWE* < 0.05), V2 (mean increase = 8.79% ± s.e.m. = 3.36%, *t*_48_ = 2.61, *PFWE* < 0.05) and V3 (mean increase = 10.95% ± s.e.m. = 3.61%, *t*_49_ = 3.03, *PFWE* < 0.05). In both conditions and for all three visual areas pRF size monotonically increased with eccentricity (Figure 1B). However, from ∼3–4 degrees eccentricity, pRFs were significantly bigger for high perceptual load at fixation; early visual cortex representations of the surrounding region were blurred when the central fixation task was higher in perceptual load. This resonates with previous findings showing that shifting the focus of *spatial* attention away from a target yields perceptual blurring [7], renders spatial information carried by the BOLD signal less precise [8] and increases the size of single neuron receptive fields in area MT [9].

RETRACTED

Apart from pRF size, perceptual load also affected pRF locations. We calculated shifts of pRF centre positions (comparing high *versus* low load) and expressed them relative to the respective pRF sizes. The average centre position of pRFs became significantly more eccentric under high load in V1 (mean = 5.92% ± s.e.m. = 2.45%, *t*_45_ = 2.41, *PFWE* < 0.05) and V3 (mean = 8.29% ± s.e.m. = 2.44%, *t*_45_ = 3.40, *PFWE* < 0.01) with a similar trend in V2 (mean = 3.81% ± s.e.m. = 2.71%, *t*_51_ = 1.41, *PFWE* = 0.17; Figure 1D). Like the blurring effect, this ‘centrifugal’ effect on pRFs was strongest from ∼3–4 degrees eccentricity. However, it showed a steep decline after a peak at ∼4–5 degrees (Figure 1D). This centrifugal effect contrasts with previous findings that neurons in, for example, LIP [10] and MT [9] shift their receptive fields *towards* the focus of attention. Interestingly, we observed such a ‘centripetal’ change of pRF eccentricity for preliminary data from IPS (the human homologue of LIP; mean = –14.03%, ± s.e.m. = 4.35%, *t*_16_ = –3.23, *PFWE* < 0.01; note that we could map IPS only for a subsample and pRF size in IPS did not change significantly; see Supplemental Figure S1J–L for details). This suggests that perceptual load at fixation induces a repulsion effect on the smaller pRFs of early visual cortex, while attracting the bigger pRFs of higher areas.

We conducted several control analyses to test the robustness of our findings. They confirmed our analyses were robust to outlier removal and were not confounded by amplitude effects, different hemodynamic profiles or eye movements (see Supplemental Figures S1 and S2).

Our findings demonstrate that increased demands on central target processing affect the representation of the surrounding visual field in early visual cortex. This representation becomes spatially coarser and pRFs are repelled centrifugally. This in turn could reflect receptive field changes at the single neuron level (for example [9]) or a differential change of amplitudes between subpopulations within a voxel. For instance, a radial gradient of load-induced amplitude suppression [1] could shift weighting within a voxel to units with larger and more peripheral receptive fields causing pRF changes similar to those we observed (c.f. Supplemental Results for a detailed discussion and control analyses addressing this possibility).

RETRACTED

A ‘blurring’ of neural representations resonates with studies investigating *spatial* attention and its effect on single unit receptive fields [9] as well as on the spread of stimulus-evoked BOLD responses [8]. Our results extend these findings by demonstrating that the spatial tuning of neuronal populations in human V1–3 is affected by perceptual load. We propose neural ‘tunnel vision’ as a form of distractor suppression under high perceptual load. Our results also add to findings regarding the attentional shift of receptive fields. Single unit receptive fields in, for example, area LIP are attracted by the focus of attention [10], an observation that has been linked to perceptual repulsion effects. We found a similar effect of central perceptual load in IPS, but at the same time pRFs in areas V1–3 were repelled by perceptual load at fixation. This demonstrates that attention can affect the spatial tuning of different neuronal populations along the visual hierarchy in opposite ways, possibly related to both the size of pRFs and their distance to the target. It also points the way to future work examining whether the relationship of these neuronal populations to perceptual effects of attention can be similarly dissociated.

We speculate that the perceptual consequences of changes in neural spatial tuning might depend on the representational properties of the neural populations involved. Specifically, spatial tuning changes might go along with perceptual mis-localisation and altered acuity for neural populations that act as ‘labelled lines’ for perception. The same changes in neural populations that can dynamically change their ‘labels’ might cause a more general re-distribution of perceptual sensitivity across the visual field.

## Supplemental Information

Document S1. Supplemental Experimental Procedures, Results and Two Figures
